The article "Combining AI Techniques for Recognizing Aerobics Sport Videos" was retracted in 2023. Reasons: signs of a paper mill; suspected computer-generated content; unreliable results or conclusions; lack of ethics approval or compliance.

# Combining AI Techniques for Recognizing Aerobics Sport Videos

**DOI:** 10.1155/2022/2293122

**Published:** 2022-06-17

**Authors:** Meiling Duan

**Affiliations:** Zhengzhou Preschool Education College, Zhengzhou 450000, China

## Abstract

In order to improve the recognition accuracy of aerobics athletes' action features, a multifeature fusion-supported aerobics footprint recognition framework was proposed in this work. By extracting and constructing the 3D peripheral structure reconstruction scheme of the concept of aerobics footprint, we combine the fuzzy feature decomposition method to decompose the aerobics footprint image with multi-pane and suggest fusion. We further realize the similarity identification of aerobics athlete's trajectory through the wear polymorphic liquefaction method. Simulation results have shown that our proposed method has better effect on the similarity recognition of bodybuilders' footprints, a higher accuracy of behavior location, a satisfactory notification time, and an accurate recognition of bodybuilders' footprints. Experiments have shown that our designed system has a small mean square error of aerobics movements and a confirmation of absolute failure. It also has a high recognition fidelity. Noticeably, the reason for the difficulty of aerobics coordination of 10 athletes and the confusion of actual coordination is small, and the accuracy of the Beer effect is high. Our method can be applied for body building, and it can provide the foundation for Game Bill.

## 1. Introduction

In aerobics competitions, referees will reason about the embarrassment of the athlete's operation according to the opponent's rules, thereby making a net valuation of competition motivation. However, in the current development of aerobics refereeing, there is a lack of a unified and random movement embarrassment scoring system. The aerobics difficulty score that you can enjoy objectively alone cannot objectively and accurately evaluate the sports performance of athletes, and the lack of fairness in recording results is controversial [1–12]. Therefore, there is an urgent need for a professional, reasonable, and standardized automatic scoring system for the difficulty of aerobics. Automatically run the cause system, and use the Bayesian best classifier for action recognition on the basis of setting up the broken graph monitoring process. The experimental question shows that the aerobics contract account is achievable, but the confirmation reliability needs to be modified. Lu Mo and others designed an auxiliary evaluation system for amusement competitions based on big data and behavior recognition algorithm rules, they established a record comparison banner database, and integrated the depth shape and skeletal features filtered by the algorithm. In order to further improve the scientificity of the recording effect of aerobics, this paper uses the action recognition algorithm to design an automatic scoring system for the difficulty of aerobics based on the behavioral attention algorithm rules. Automatically evaluate the action test, clarify the standardization, offering and scientificization of aerobics obstacle charges, and promote the sustainable development of aerobics.

The prosecution of aerobics stirring images ordered the use of the idol push method, and the shape analysis and recognition ability of the aerobics stirring copy was not recognized. Research into the discovery method of aerobics flight screen, which can correct and optimize the movement of the athlete. The generation and notification of the image is based on the establishment of the image target peripheral detection and division model, the three-dimensional feature amount pedigree of the aerobics athlete's trajectory similarity, combined with the image form to complete the aerobics abdominal muscle image notification [1]. Footprint image recognition method is of great significance to the movement analysis and correction of aerobics athletes. Reference [2] discussed an adaptable notice sequence of aerobics decomposition operation show based on morphological lineage. The basic subtraction method extracts the hominine strength target of aerobics, holds the double star composition of the outline of the humanoid splendor, and prevails the aspect rate of the rectangular beyond the contour. Gender discovery matching decompounded treatment actors are recognized and dissolved into shape, a similarity threshold is set, and the charismatic similarity is higher than the gate when identification is terminated. The accuracy rate is extremely high, and the recognition time is prolonged. Aiming at the above problems, this paper proposes a verification rule for aerobics athletes' footprint replication based on multifeature fusion. Firstly, an image acquisition mode of aerobics footprints is constructed, and then three-dimensional shape reconstruction and feature descent are performed on the images. Combined with the method of multidimensional shape liquefaction, the bodybuilder's hamstring copy notification is networked, and the simulation experiment analysis is completely launched, which reveals the superior performance of this method in improving the bodybuilder's trace appearance recognition ability.

In order to solve the problem of poor robustness of confirmation results caused by the gentle tilt of the old method due to factors such as motion cost, lighting conditions, closure, and composite background, an adaptive confirmation problem of aerobics decomposition posture is proposed to be studied by a feature extraction system. The video sequence is divided into several body segments by time-efficiency mounts, and the result is not all aerobic exercise, but an accident that interferes with intelligence. Using the canine distemper subtraction rule, the human body target is lowered for aerobics exercises, and further protrusions are performed to obtain the outline of the human body. Get the ratio of the width and height of the outer contour of the rectangle, get the ladder diagram according to the view scale, and use the Laplace method to explain the light flooding between adjacent difference frames to reduce the prestige of background clutter. The shape vector is extracted from the key frame, and the bodybuilding decomposition action image to be yielded is matched with the extracted features through parity perception, and the parity starts to be adaptive. An illustration of our designed aerobics recognition system is shown in Figure 1.

## 2. Related Work

It is true that some people are in a state of health and more and more society is focusing on therapeutic exercise. Aerobics is a relatively shallow and popular sport that has been receiving extensive attention [1, 2]. Decomposition teaching is the essential content in the process of aerobics education, and the realization of decomposing action image recognition directly affects the expression of aerobics teaching. Therefore, it is of great significance to study an effective method for self-adaptive confirmation of the concept of aerobics disintegration movements [3, 4]. There are many factors affecting the recognition performance of traditional methods, such as direct rate, brightness, occlusion, and complexity, and the robustness is poor [5]. Therefore, a new method is proposed to solve this problem, which assembles the decomposed action image samples of aerobic exercise into open boxes, makes their shape drop, and realizes the adaptive recognition of dissolved action images through feature similarity replication.

The dynamic system configuration of the aerobics obstacle robot based on the behavior confirmation algorithm program is shown in Figure 1. System configuration includes data gain layer, communication layer [10–14], data bulge layer, and nickname boost. The ram component in the data acquisition lift is the somatosensory sensor Kinect, which uses the somatosensory Kinect extensively to obtain the somatosensory enlightenment of bodybuilders and obtain proxy images of bodybuilders [5, 6]. The built-in aerobics gesture performance is transmitted to the data growth bed through the communication protocol; the data bony protuberance layer uses the largest pro-chrono continuum. The random access memory function of the application layer is the robot score against the aerobic exercise; it is powerful The Aerobic Impairment Score–based test automatically earns the Aerobic Embarrassment Score. Somatosensory Sensor Kinect Kinect is a 3D somatosensory sensor, which can teach energy about the retention degree of the network [9, 10]. The construction of the somatosensory Kinect is shown in Figure 2. Somatosensory Kinect has focus tracking technology, and the underlying engine rotates with the movement of aerobics. The infrared transmitter projects an optical maser that cannot be recognized by Christian eyes to the aerobics, then obtains the position and emotional complaints of the aerobics through the infrared camera, and outputs the action images of the aerobics idler through the species camera [13–16].

The multidimensional periodic thread of aerobics' fighting stance is conditioned because this sequence depicts an honest calisthenics gesture and spatial sensory data. The action data that runs as n in the jth scope is set to aj. Due to variation in aerobics movements, similar conditioning of the same activity is not 100% consistent, so movement data must be normalized to eliminate this variance [11]. For the j-dimensional time series aj of the calisthenics concept, its normalized mode is to remove noise interference and overcome seasonal depletion. It can further use symbol aggregation to convert aerobic spread-delay sequences into separated symbol sequences. Using the piecewise aggregation approximation technique, the age sequence of aerobics figures is divided into line segments of the same size.

Redundant algorithms based on the highest analogy-leas can filter and populate different examples and wealth of calisthenics movement features. The selection step is divided into two steps: (1) Use the feature reference algorithm ReliefF to evaluate the unique performance of each aerobics movement form and conform to the aerobics movement characteristics and express. Relevance is used to plan feature weights, and the aerobics operation features that affect less than the threshold *ε* will be discarded, and the features with strong family reciprocity are selected as candidate features. (2) Distinguish the correlation between authorization forms and leaves. ReliefF algorithm rules are more useful in the feature selection proposition in the flag problem. It can identify weights for each bodybuilding action feature in weakly multiple iterations. In the repeated process, the ReliefF algorithm is all in the aerobics movement data. A trypiece Z is randomly selected from the set, and k-next-neighbor patterns are obtained in the same type. There are two modes of shape union and feature redundancy in the supervisor feature. In practical applications, too many license shapes must be removed. Therefore, according to the influence, the action features are descendants, and the aerobics action features below the threshold are removed.

## 3. Our Proposed Method

The form of the automatic scoring system for aerobics difficulty supported by the action confirmation algorithm program is shown in Figure 1. The system builds rake data access layer, communication layer, data processing layer, and ointment response layer. The assembly component in the data acquisition bed is the somatosensory sensor Kinect, which mainly uses the somatosensory sensor Kinect to collect the bodybuilder's somatosensory instructions and obtain the bodybuilder's action images [5, 6]. Pass the collected aerobics action concept to the second-hand connection program of the data processing layer; the data processing base adopts the maximum correlation-minimum redundancy contact layer combination function to automatically record the embarrassment of aerobics, mainly supports the difficulty standard of aerobics, and automatically realizes bodybuilding difficulty rating. The Somatosensory Kinect Kinect is a 3D somatosensory, which can realize the capture of humanistic work information [9, 10]. The structure of the somatosensory sensor Kinect is shown in Figure 2. The somatosensory sensor Kinect has a focus tracking technology, and the low-profile motor rotates with the reversal of aerobic exercise. The infrared transmitter emits the laser Rosicrucian to the human eye to the aerobics, then uses the infrared camera to obtain the aerobics posture teaching, and generates the aerobics action picture through the disguised camera.

The multidimensional time series of aerobics action pictures are set as r = r1, r2, ⋯, rm {}; this sequel represents a single aerobics action and dimensional sensor data. The behavior data of extent n in the jth extension is adjusted to aj. Because aerobics movements are contested, the same movements like prepare are not 100% compatible, so evolutionary data must be regularized to eliminate this difference [11]. For the j-dimension period scale of the inversion image of aerobics, aj, and other words, the normalization rule is

(1) $$\begin{array}{c} \eta \left(t\right)=\frac{w\left(t\right)}{a\left(k\right)+c}, \end{array}$$

where a(j) is the normalized j-dimension time sequence.

(2) $$\begin{array}{c} Q_{m}=s_{m}\left(i,j,u,v\right)+\eta \left(t\right), \end{array}$$

In the system-level disorder and decrease delay conquest, the symbol aggregation method technique is an interest to morph unbroken seasonal arrangement Aerobics test into disjunct emblem consequence. Using the piecewise aggregate course technique, the tempo series of aerobic task is divided into lobes of equal greatness [12, 13]. Under the condition of Gaussian distribution with the same likelihood, the breakpoints *C* = {*C*1, *C*2, ⋯, *Cq*} divide the exercise data interval of aerobics into q +1 segments and at the same time convert all segments into ideographic descriptions. For an age sequence aj, the number of breakpoints is q, the inclusion of segments is g, the sequence of symbols is rtj, and the sequel of flags is rtj. Each element conforms to rt j ∈ {W1, W2, ⋯, Wq + 1}, where Wq + 1 is the sign of the number of break points q + 1 in the aerobics operation picture.

DTW belongs to the frequent difference measurement mode of similarity conjectures on time scales. The two symbols run are rtx and rty, respectively, and their drop check reserves are as follows: In the formula, the lengths of a and b in the aerobic exercise evolution data are na and nb in turn. The measure of the player's action data is aj, and bj is the Euclidean distance between aerobics action data. C_min_{a, b} are the highest and lowest breakpoints of the j-th dimension aerobic exercise data aj and bj, respectively. The Euclidean divergence is a habit to measure the similarity of twin (former names) aj and bj:

(3) $$\begin{array}{c} E\left(i,j\right)=\sum t+a+\eta , \end{array}$$

The data item of aerobic exercise is the three-dimensional data in every power. Depending on the relationship between other reaches, you can determine the importance of each match. Both dual (nominal) modes can be applied. In order to obtain different aerobics behavioral characteristics, the aerobics behavioral characteristics are relatively Ga and Gb. Ga is more important for the idea of cardio.

Based on the limit correlation-minimum redundancy algorithm program, different types and guaranteed aerobic movement characteristics can be screened out. The quoting steps are digitized into two footprints: (1) The feature selection algorithm ReliefF is used to evaluate feature generation for each aerobics combat feature. Calculate the severity and category correlation of bodybuilding action features, discard bodybuilding action forms with lower impact than abutment *ε*, and select features with entity type analogy as candidate forms.

## 4. Experimental Results and Analysis

In the experiment, the aerobics analysis gesture database and the simple aerobics decomposition action database were selected as the research database, which were recorded as database A and database B, respectively, in the application. Database A has 120 aerobics videos, and there are 10 aerobics movements in the videos, which are realized by 12 aerobics athletes in the application. This dataset is Scots in a real environment, contains lighting information, and has biased obstacles. Database B stores 15 action types of aerobics, and consists of 65 videos. The video resolution of both databases is 720 pixels ×480 pixels, and the degree is 80 frames/second. Figure 2 explains the aerobics decomposition action idols in part A of the database, and Figure 3 guides the aerobics decomposition action images in part B of the database. It should be noted that database A has different scenes, the end of survival dilemma changes, family scenes, outdoor scenes, etc. The pictures registered below are all real aerobics analysis actions; in addition, it also contains a lot of interference pictures. For the convenience of analysis, we first test the litmus test on the database management system B. Block A bodybuilding decomposition action in DBMS B was forcibly selected and analyzed using this newspaper process, glossy scholarship course, and hierarchical time recall method. The analysis of Figure 4 shows that the course in this paper has the most accurate notification problem for the decomposition of aerobics demeanor and can effectively identify aerobics' multiple decomposing movements. However, there are real errors in the recognition of word-based scientific patterns and the hierarchical time recall method, indicating that the accuracy of regularity recognition in this paper is high. In order to further verify the notification accuracy of the method in this paper, the raise-one-out peevish-validation rule is used to prove that in each round of experiments, the legacy action is the habit of managing data. Identify the confusion matrix. Figure 3 shows the informed confusion matrix, vocabulary learning pattern, and hierarchical transient memory pattern of database B of our method. From the analysis, it can be seen that the process of this paper is used to identify the decomposing actions of aerobics. Only the two decomposing actions of trunk transection and pacing undoubtedly have recognition errors and confusion events, and the recognition results of other actions are relatively accurate.

The following is the hierarchical temporary storage method of the notification confusion array plant and the database management system B of the dictionary scientific means. Comparing Figures 3 and 4, it is found that the method in this literary has the last effect of aerobics decomposition battle in the confused position in the identification. The glossy lore method confuses the chest intersection gesticulation with fisticuffs, honest fighting, bow saccharine movement, and movement mechanism. The memory process scattered and accumulated oblique movements along with fist movements, foot movements, and footprint movements, and the degree of confounding was higher than that in this paper. 2.3 Recognition effect of database A In order to further reflect the effectiveness , this paper uses dictionary lore method and hierarchical time memory method to identify the habit of aerobics decomposition action in database management system. The three methods are habits in different scenarios.  Table 1 describes the results of the description of notification accuracy. From the analysis in Table 1, it can be seen that in database B, the attention accuracy of the three methods for low-light scenes and outdoor scenes is relatively moderate, while the attention accuracy for intra-wall scenes is relatively high. The notification accuracy rate of different scenarios is high, which further affirms the accuracy of the method in this paper.

In order to verify the required performance of this publication's process in realizing the bodybuilder's pug image notification, a simulation experiment was carried out. Attempts are intended by Matlab 36. The length of the dividing line is 12, the number of sampling samples for the concept of aerobics footprint is 200, the sampling population of the three-dimensional visual feature of the image is 24 kHz, and the range appearance of a single design conforms to the 1024 standard. According to the above parameter settings, the step recognition of aerobics athletes is completed, and the original idol is shown in Figure 3. The original picture of aerobics in Figure 1 is denoised, and the production result is shown in Figure 3. The analysis of Figure 3 shows that the regularity of this paper can be powerfully obtained. On this basis, the facial contour features.

In order to judge the general introduction of the system in this paper, Matlab software is used to measure and calculate the system scheme, and the system running platform is Windows XP. The sampling population of aerobics moving images is 650 × 490, and the system in this paper is a necessary condition for reasoning about the difficulty of aerobics against exercise. According to the 2017-2020 aerobics competition rules, it can be seen that the obstacle standards of dynamic support movements, stable and robust movements, bouncing movements, and balance and flexible movements in aerobics competitions. The action data are shown in Table 1. The mean square error (MSE) and mean infinite irregularity (MAE) of the system in different four groups of aerobic exercise were tested. The calculation methods of MSE and MAE are as follows: *n* is the number of aerobic exercise confirmations; *i* is the matching amount of aerobic exercise behavior confirmation; e^i and ei are the count of avow actions and a certain number of actions, respectively. The negligible absolute errors representing regular hallucinations and discriminative reasoning are negligible compared to jumping, balancing, and pliable movements, with a limit utility of no more than 0.02 (Figure 4). The confirmation accuracy rate is high, and it has a positive performance on the perplexity description of subsequent actions.

In the preparation of data thanks to the Kinect Humane Agency, the aerobic exercise data of 10 athletes were randomly cited, and the aerobic exercise data of 10 athletes was the automatic power wearing system in this paper. The rational utility of the perplexity coefficient and the extreme competition of actively opposing cooperation are 0.1, and the out-of-bounds value is weak and within an acceptable range. In this paper, when evaluating trials of aerobic exercise, only athlete size 4 performed the senhorita, while Mademoiselle had a number of 1, and the desired number of movements was relatively small. There are many purposes of error evaluation, such as nonstandard movements of athletes, which causes the system to filter it out very quickly when doing action recognition, which has no serious impact on the counting results of this fictitious system, and a charge rise is possible. The 3D optical reconstruction and feature drop of calisthenics footprints using the sequence in this paper has higher accuracy and better recognition performance. In the process of causality identification, the garnet model of 6,000 bodybuilders was calibrated and analyzed using the course and literature [2] system of this newspaper, and the peak memory-to-noise ratio was compared between the two methods. The analysis of the above process shows that the peak signal-to-noise ratio of the method in this paper is 23.22 dB higher than that of the learned [2] mode; its site fidelity is 11.33% higher than that of the belles-lettres [12] method; its recognition speed is higher than that of the literature [15] The recognition time is 2.69 s shorter. It is shown that the method in this example can completely realize the portrait notification of aerobics' footprints, correct the positioning ability of the action, and reduce the confirmation delay of the action performance. Since the sequence in this paper adopts the accumulation of the three-dimensional form, the three-dimensional reconstruction of the footprints of the bodybuilder is implied, thereby improving the body shape correction ability of aerobics.

## 5. Conclusions

Aiming at the problems of the unwritten aerobics champion track similarity prompt method, which has problems such as large delay in notification of action similarity and high authenticity of action positioning, which leads to poor recognition performance, a multiform joint support concept of gunpowder for aerobics and acrobats is designed. I am interested in the image acquisition design of the foot trajectory and the edge contour feature generation system to reduce the low-level behavior of the aerobics footprint image, and design a three-dimensional surrounding structure reconstruction model of the aerobics footprint display. Multi-ladder analysis and information fusion are the winners, and the polymorphic combination method is a habit to realize the similarity recognition of bodybuilders' footprints. Research reflected that notifications of images of aerobics footprints in the class are customized. It will reduce confirmation opportunity overhead.

## Figures and Tables

**Figure 1:** the pipeline of our proposed aerobics sports recognition system.

**Figure 2:** Examples of Kinect data from aerobics sports.

**Figure 3:** Confusion matrix of different aerobics sport actions.

**Figure 4:** Performance on different athletes.

**Table 1:** Comparison of three aerobics sport actions recognition algorithms.

Method	Lighting	Indoor	Outdoor	Average
Text	91.213%	95.436%	87.695%	90.324%
Dictionary	83.445%	89.443%	79.546%	85.456%
Hierarchical	86.576%	91.324%	80.435%	86.780%

## Data Availability

The data used to support the findings of this study are available from the corresponding author upon request.
